This article has been retracted.

# Analysis of Clinical Efficacy of Laparoendoscopic Single-Site Surgery for Uterine Fibroids

**DOI:** 10.1155/2022/5606998

**Published:** 2022-04-11

**Authors:** Wei Zhu, Shiqin Mao, Yan Chen, Xiang Kong

**Affiliations:** ^1^Medical College, Yangzhou Uniersity, Yangzhou 225001, China; ^2^Deparment of Gynecology, People's Hospital of Jingjiang, Jingjiang 214500, China; ^3^Institute of Translational Medicine Medical College, Yangzhou University, Yangzhou 225001, China; ^4^Jiangsu Key Laboratory of Experimental & Translational Non-coding RNA Research, Yangzhou 225001, China; ^5^Department of Obstetrics and Gynecology Clinical Medical College, Yangzhou University, Yangzhou 225001, China

## Abstract

In order to determine the clinical efficacy of laparoendoscopic single-site surgery (LESS) for uterine fibroids (UFs), the study population comprises 65 patients who underwent hysteromyoma enucleation in our hospital from January 2020 to September 2021. Among them, 30 patients with conventional multiport laparoscopic myomectomy (MLS-M) are taken as the control group (CG), and the rest 35 patients with laparoendoscopic single-site myomectomy (LESS-M) are taken as the research group (RG). Perioperative indicators and incidence of complications are compared between groups. Measurements of inflammatory factors (IFs) (tumor necrosis factor (TNF)-*α*, interleukin (IL)-6, and C-reactive protein (CRP)) as well as ovarian function indices (follicle stimulating hormone (FSH), luteinizing hormone (LH), and estradiol (E2)) were carried out by using ELISA. Patients' pain sensation, body image satisfaction, incision aesthetic satisfaction, and quality of life (QOL) are assessed using the Visual Analogue Scale (VAS), Body Image Scale (BIS), Cosmetic Score (CS), and SF-36, respectively. LESS-M is beneficial to patients' early recovery after operation, with little influence on ovarian function and high incision aesthetic satisfaction, which reserves clinical popularization.

## 1. Introduction

Uterine fibroids (UFs), the most common benign tumor in the uterus, present an incidence of about 60% in fertile women [1]. Although most women with UFs are asymptomatic, approximately 30% will develop serious symptoms, such as anemia, emmeniopathy, sterility, constipation, metrorrhagia, and abortion [2]. Surgical resection is currently the main means of clinical treatment for this disease, among which traditional laparotomy has been gradually phased out due to the disadvantages of large trauma and multiple complications [3]. Laparoscopic myomectomy, in virtue of small incision, few complications, and fast recovery, has emerged as the constant development of laparoscopic technology and has been gradually applied to the clinical treatment of UFs, which can promote the early recovery of patients [4]. At this stage, multiport laparoscopic myomectomy (MLS-M) is mainly used in clinical practice. However, with the deepening of the concept of minimally invasive surgery, many young patients are not only satisfied with retaining fertility, but also pursuing cosmetic needs [5]. Today, laparoendoscopic single-site myomectomy (LESS-M) is increasingly concerned, as it is less invasive than conventional three- and four-port surgery, which is conducive to patients' rapid recovery with better cosmetic effects [6, 7]. However, there is currently a paucity of comparative studies on LESS-M and MLS-M in patients with UFs, resulting in the insufficiency of evidence-based medicine evidence for its application effect and safety in the disease. Consequently, this paper discusses the clinical efficacy and safety of the above two procedures applied to UFs, aiming at finding out the most feasible and suitable surgical approach for UF patients.

The study population comprised 65 patients who underwent hysteromyoma enucleation in our hospital from January 2020 to September 2021, including 30 cases (control group, CG) with conventional multiport laparoscopic surgery (MLS), and 35 cases (research group, RG) with LESS. The inclusion criteria were as follows: diagnosis of UFs by preoperative ultrasonography, MRI, and hysteroscopy; the American Anesthesia Association (ASA) classification ≤ Grade II; and no operative contraindications. The exclusion criteria were as follows: body mass index (BMI) ≥ 30 kg/m^2^; coagulation dysfunction or taking drugs that may affect coagulation function within 3 months prior to enrollment; complicated with gynecological inflammation such as chronic pelvic inflammatory disease and vaginitis; use of hormone drugs within 3 months of enrollment; obvious surgical scar in lower abdomen; and those unable to cooperate with all evaluations.

## 2. Surgical Procedures

Both groups of patients are operated by the same group of surgeons, who are skilled and cooperated well. Preoperative preparation and postoperative treatment are basically the same.

Patients in CG are treated with MLS-M: patients are placed in the supine position with a longitudinal incision 10 mm below the umbilicus as an observation hole, and the laparoscopy is inserted. A 10 mm incision is then made via the reverse McBurney as the operation hole, and the puncture trocar is placed. Thereafter, a 5 mm incision is created at the intersection of the right paramidline and 20 mm above the pubic symphysis as an auxiliary operation hole, and a puncture catheter is placed. A CO_2_ pneumoperitoneum is established through this incision, and the pneumoperitoneum pressure is maintained at 12–14 mmHg. The abdominopelvic cavity is carefully investigated by laparoscopy, and instruments such as forceps are placed to separate and remove the myoma lesions under the microscope. Active bleeding sites are treated with bipolar electrocoagulation or 8-shaped suture fixation for hemostasis, followed by suture with absorbable sutures. The removed tumor tissue is put into the extraction bag and removed from the umbilical region. Finally, the umbilical incision is reshaped and closed with absorbable sutures.

Patients in RG are treated with LESS-M: patients are placed in the position of head low and feet high, about 15°, and a 20 mm longitudinal incision is made through the midline of the umbilicus to establish a CO_2_ pneumoperitoneum. Under direct vision, the single-port multichannel cannula is placed into the abdominal cavity through the guide, and after unloading by the guide, the single-hole multichannel cannula and its outer ring are fully fixed. Then, a laparoscopic probe is placed to explore the abdominopelvic cavity under the microscope, and surgical instruments are placed. During the operation, conventional laparoscopic surgical instruments or lengthened instruments are used to complete the operation. The serosa and muscular layers are longitudinally incised with a monopolar electric hook. Microscopically, the UFs are pulled by claw forceps and separated along the pseudocapsule to completely remove the fibroids. Active bleeding sites are stopped by bipolar electrocoagulation or 8-shaped suture fixation, and the rest of the operations are the same as in the control group.

Perioperative indicators and complications of the two groups are recorded. The former included intraoperative blood loss (IBL), operation time (OT), the first postoperative anal exhaust, early ambulation, and length of stay (LOS), while the latter included common complications such as incision infection, pelvic adhesions, and adhesive intestinal obstruction.

For the detection of inflammatory stress factors, peripheral venous blood (3 ml) is sampled from each patient 1 day before the operation, as well as 1 day and 1 month postoperatively, and centrifuged (1,000 × g, 4°C) for 15 min to obtain the supernatant. Measurements of inflammatory stress factors (tumor necrosis factor (TNF)-*α*, interleukin (IL)-6, and C-reactive protein (CRP)) and ovarian function indexes (follicle stimulating hormone (FSH), luteinizing hormone (LH), and estradiol (E2)) were carried out by adopting enzyme-linked immunosorbent assay (ELISA) with ELISA kits all supplied by Abcam, USA.

Patients' pain is assessed one day after surgery using the Visual Analogue Scale (VAS) [8]. The scores ranged from 0 to 10, with higher scores indicating intense pain. At one month postoperatively, patients' physical satisfaction is evaluated with the Body Image Scale (BIS) [9] (score range: 5–20). The higher the score, the more satisfied they are with their physical condition. The incision aesthetic satisfaction of patients is evaluated with the Cosmetic score (CS) [9]. With a score ranging from 3 to 24 points, the score is positively associated with satisfaction with the incision aesthetic.

Thirty days after surgery, patients' QOL is evaluated via the Short-Form 36 Item Health Survey (SF-36) [10], involving five evaluation items (social function, physiological function, emotional function, mental health, and bodily pain). The total score of each item is 100 points, and the score is proportional to the patient's QOL.

The data collected are subjected to statistical processing and visualization using SPSS 22.0 and GraphPad Prism 6, respectively. For the comparison of count data, the Chi-square test or Fisher exact test is used. For measurement data, the differences between groups, within the group before and after surgery, as well as among multiple groups are performed using independent *t*-test, paired *T*-test, as well as one-way ANOVA plus post hoc verification, with *P* < 0.05 representing statistical significance.

## 3. The Experimental Results

### 3.1. General Information

RG and CG showed no comparable general information such as age, BMI, number of fibroids, diameter of fibroids, course of disease, histological type, marital status, residence, and educational background (*P* > 0.05).  Table 1 shows the comparison of general information.

### 3.2. Perioperative Indicators

Surgery is successfully completed in both groups, with no cases of conversion to laparotomy or an increase of puncture holes. The IBL and OT differed significantly between groups (*P* > 0.05). However, earlier postoperative anal exhaust and ambulation, as well as shorter LOS, are determined in RG (*P* < 0.05).  Table 2 shows perioperative indicators.

## 4. Occurrence of Complications

The number of cases of incision infection and pelvic adhesions in RG is 1 and 2, respectively, with a total incidence rate of 8.57% (3/35). In CG, incision infection occurred in 2 cases and pelvic adhesions in 3 cases, with a total incidence of 10.00% (3/30). The two arms showed no statistical difference in the complication rate (*P* > 0.05).

### 4.1. Comparison of Inflammatory Stress Factor Levels

ELISA showed no evident differences in preoperative CRP, TNF-*α*, and IL-6 levels between groups (*P* > 0.05). Postoperatively, CRP, TNF-*α*, and IL-6 elevated in both arms and are lower in RG (*P* < 0.05).  Figure 1 displays a comparison of inflammatory stress factors.

### 4.2. Comparison of Ovarian Function

ELISA identified no statistical differences in preoperative E2, FSH, and LH between groups (*P* > 0.05). In both arms, E2 declined while FSH and LH increased statistically after surgery (*P* < 0.05). And compared with CG, E2 is lower while FSH and LH are higher in RG (*P* < 0.05).  Figure 2 shows the comparison of levels of ovarian function-related indicators.

### 4.3. Comparison of Postoperative Pain as well as Body Image and Incision Aesthetic Satisfaction

Statistically, RG exhibited a lower VAS score one day after surgery than CG, and higher BIS and CS scores at one month postoperatively (*P* < 0.05).  Figure 3 shows the comparison of postoperative pain, as well as body image and incision aesthetic satisfaction.

### 4.4. Comparison of QOL

The evaluation of patients' QOL one month after operation revealed significantly higher scores of social function, physiological function, emotional function, mental health, and bodily pain in RG versus CG (*P* < 0.05).  Figure 4 displays the comparison of patients' quality of life 1 month after surgery.

QOL, as people's living quality and medical level constantly improve, is also considered as the evaluation standard of treatment efficacy. There are many factors influencing the QOL of female surgical patients, among which pain and body satisfaction are the major factors. Our results identified earlier first postoperative anal exhaust and ambulation, as well as shorter LOS in RG compared with CG. In addition, RG showed a notably lower VAS on the 1st day after the operation and higher BIS, CS, and SF-36 scores at one month postoperatively. It suggests that LESS-M is less traumatic and can validly enhance the postoperative QOL of patients with UFs. The reason is that there is only one incision in the LESS-M, which reduces surgical trauma and consequently leads to milder postoperative pain; moreover, the natural depression of the umbilical part can play a role in hiding the scar of the incision.

Through the upregulation of tissue trauma, pain perception, and psychological factors, the hypothalamic-pituitary-adrenal axis and sympathetic nervous system can be activated to trigger the stress response; moreover, the hypothalamus stimulates the release and production of hormones from the pituitary gland and the increase of a variety of inflammatory cytokines, which aggravates the stress response to surgery. Evidence has shown that strong inflammatory stress is not conducive to the postoperative rehabilitation of patients. CRP, TNF-*α*, and IL-6 are common inflammatory cytokines, and their levels increase with the severity of inflammation. In our research, the postoperative CRP, TNF-*α* and IL-6 levels are elevated markedly in both arms, but are lower in RG versus CG, further demonstrating that LESS-M has less trauma and traumatic stress reaction, which is more conducive to patients' postoperative rehabilitation. Preserving fertility is one of the main demands of fertile women for surgical treatment of UFs. The ovary is a vital organ for women, with reproductive function and endocrine regulation function. However, myomectomy has a negative impact on ovarian function due to the trauma to the patient's uterus. FSH, LH, and E2 are critical indices for clinical evaluation of ovarian function. Our results showed reduced E2 and elevated FSH and LH in both arms after the operation. And compared with CG, E2 is lower while FSH and LH are higher in RG. This also suggests that the LESS-M is less harmful to the patient's body.

## 5. Conclusion

This paper still shows some margins of improvement. First, there is no long-term follow-up of patients due to limited time, so it is not known whether there is a significant difference in the follow-up recurrence rate and the pregnancy rate between the two surgical procedures. Second, over the past few decades, the number of women who deliberately delay pregnancy has increased, resulting in an increasing number of patients over 40 with UFs. Given that patients enrolled are mainly between 20 and 40 years old, we hope to enrich our results by studying patients over 40 years old in the subsequent research.

To sum up, LESS-M is more advantageous over MLS-M for the treatment of UFs and deserves to be popularized and applied clinically because it causes less physical damage to patients, with the ability to promote patients' postoperative recovery, reduce postoperative pain, and improve QOL and surgical satisfaction.

## Figures and Tables

**Figure 1:** Comparison of inflammatory stress factors: (a) comparison of serum CRP levels; (b) comparison of serum TNF-*α* levels; and (c) comparison of serum IL-6 levels.

**Figure 2:** Comparison of levels of ovarian function related indicators: (a) comparison of serum *E*_2_ levels; (b) comparison of serum FSH levels; and (c) comparison of serum LH level.

**Figure 3:** Comparison of postoperative pain as well as body image and incision aesthetic satisfaction: (a) comparison of VAS scores 1d after surgery; (b) comparison of BIS scores 1 month after surgery; and (c) comparison of CS scores 1 month after surgery.

**Figure 4:** Comparison of patients' quality of life 1 month after surgery: (a) comparison of social function scores one month after operation; (b) comparison of physiological function scores one month after operation; (c) comparison of emotional function scores one month after operation; (d) comparison of mental health scores one month after operation; and (e) comparison of bodily pain scores one month after operation.

**Table 1:** Comparison of general information.

Groups	Control group (*n* = 30)	Research group (*n* = 35)	*χ* ^2^/*t*	*P*
Age (years)	28.60 ± 4.60	29.26 ± 5.18	0.539	0.592
BMI (kg/m^2^)	22.98 ± 1.45	23.10 ± 1.64	0.310	0.758
Number of fibroids	2.83 ± 1.39	2.74 ± 1.27	0.273	0.786
Maximum diameter (cm)	5.88 ± 1.69	5.64 ± 1.57	0.593	0.555
Course of disease (month)	10.07 ± 4.02	9.31 ± 3.79	0.784	0.436
Histological type			0.198	0.656
Intramural myoma	19 (63.33)	24 (68.57)		
Subserous myoma	11 (36.67)	11 (31.43)		
Marital status			0.002	0.964
Married	23 (76.67)	27 (77.14)		
Single	7 (23.33)	8 (22.86)		
Residence			1.233	0.267
Rural	13 (43.33)	20 (57.14)		
Urban	17 (56.67)	15 (42.86)		
Educational background			0.002	0.968
≤Junior high school	19 (63.33)	22 (62.86)		
>Junior high school	11 (36.67)	13 (37.14)		

**Table 2:** Perioperative indicators.

Groups	Control group (*n* = 30)	Research group (*n* = 35)	*χ* ^2^/*t*	*P*
Intraoperative blood loss (mL)	63.93 ± 12.20	65.91 ± 11.53	0.672	0.504
Operation time (min)	62.33 ± 8.29	64.51 ± 8.49	1.043	0.301
First anal exhaust time after operation (h)	14.87 ± 3.32	10.74 ± 3.0	5.267	<0.001
First ambulation after operation (h)	7.67 ± 3.20	5.46 ± 2.84	2.950	0.005
Length of stay (d)	6.37 ± 1.92	5.09 ± 2.12	2.534	0.014

## Data Availability

The data used to support the findings of this study are available from the corresponding author upon request.
